# Influence of “Hospital-Community-Family” Integrated Management on Blood Pressure, Quality of Life, Anxiety and Depression in Hypertensive Patients

**DOI:** 10.1155/2022/1962475

**Published:** 2022-10-04

**Authors:** Wanzhe Shi, Lei Cheng, Yang Li

**Affiliations:** Department of Cardiovascular Medicine, First Affiliated Hospital of Baotou Medical College, Baotou, Inner Mongolia 014010, China

## Abstract

**Objective:**

To explore the Influence of “hospital-community-family” integrated management on blood pressure, quality of life, anxiety and depression in hypertensive patients.

**Methods:**

A total of 60 patients with hypertension were treated in our hospital from July 2019 to July 2021. The patients were randomly divided into control group (n =30) and study group (n =30). The former accepts routine management, while the latter accepts “hospital-community-family” integrated management. Nursing satisfaction, blood pressure, disease awareness rate, anxiety and depression scores, disease control ability and quality of life scores were compared.

**Results:**

First of all, we compared the nursing satisfaction: the study group was very satisfied in 25 cases, satisfactory in 4 cases, general in 1 case, the satisfaction rate was 100.00%, while in the control group, 10 cases were very satisfied, 8 cases were satisfied, 7 cases were general, and 5 cases were dissatisfied, the satisfaction rate was 83.33%; The nursing satisfaction of the study group was higher than that of the control group (P <0.05). Secondly, we compared the level of blood pressure. There was no significant difference before management (P >0.05) but the blood pressure decreased after treatment. In the control group, the level of blood pressure in the study group was lower than that in the control group (P <0.05). In terms of disease awareness rate the scores of hypertension related knowledge hypertension harmfulness community management methods regular reexamination and blood pressure monitoring in the study group were significantly higher than those in the control group (P <0.05). There was no significant difference in anxiety and depression scores before treatment (P >0.05), but decreased after treatment. Compared with the control group, the anxiety and depression scores of the study group were lower (P <0.05). In terms of disease control ability, the total scores of diet management, medication management, behavior management and information management in the study group were higher compared to the control group (P <0.05). Finally, we compared the scores of qualities of life. Before management, there exhibited no significant difference (P >0.05). After management, the scores of quality of life decreased. Compared to the control group, the scores of physiological function, psychological function, social function and health self-cognition in the study group were lower than those in control group (P <0.05).

**Conclusion:**

The application of integrated “hospital, community and family” management can vertically integrate medical resources and establish a truly effective hierarchical treatment model. Integrated “hospital-community-family” management can improve patient compliance with treatment, enhance patients' self-management ability and confidence, and improve the management efficiency of medical staff.

## 1. Introduction

Hypertension is a common and frequently occurring disease among Chinese residents [1]. The results of epidemiological investigation indicate that the number of people suffering from hypertension in the world is more than 1 billion, and it is expected that the number of cases will reach 1.55 billion in 10 years' time. According to the latest hypertension guidelines in China, the prevalence of hypertension among adult residents in China is 27.9%, that is, one-third of adults suffer from hypertension, and the prevalence of hypertension in large and medium-sized cities is relatively high [2]. Cardiovascular and cerebrovascular diseases are caused, and the resulting medical expenses are also increasing year by year [3]. How to control blood pressure within the standard range to reduce complications, reduce medical costs, and improve quality of life has always been the focus of our research [4]. The data indicate that the control rate of blood pressure in adult patients with hypertension is only 16.8%. An effective model of hypertension management is needed to improve patient adherence, control blood pressure and reduce complications [5]. At present, the management of hypertension in community include health education, family intervention, community intervention, self-management and individual intervention. The above management model will make patients aware of the importance of regular medication and knowledge about hypertension, which will help to lower their blood pressure levels and thus improve their blood pressure control rate. However, due to differences in each patient's cultural and educational background, personality and family conditions, there is also variability in patient acceptance, making it difficult to effectively control the blood pressure levels of all patients [6]. Previous studies have indicated that the etiology of patients with hypertension is complex, there are significant differences in the severity of the disease, the pertinence of traditional education is not strong, not combined with behavioral intervention, so that routine management is of little significance to effectively enhance patient compliance [7]. Therefore, it is particularly important to promote the understanding of hypertension, explore scientific, effective and standardized management models, and control the development of hypertension.

At present, the existing hypertension management in China mainly includes continuous nursing, home follow-up nursing, path-based comprehensive nursing, and file management intervention mode [8]. The management mode is relatively simple, mainly in tertiary hospitals. Medical staff lack time and energy, and the continuous care provided is limited. Hospital and community management are out of touch, patients are not within the jurisdiction of hospitals or community health institutions after discharge, lack of continuous and comprehensive education and supervision, and the management compliance of patients with hypertension is far lower compared to other chronic diseases [9]. In 2009, the opinions of the CPC Central Committee and the State Council on deepening the Reform of the Medical and Health system pointed out that it is necessary to speed up the construction of a health service system based on community health services, guide general diagnosis and treatment at the grass-roots level, and gradually achieve community first treatment, two-way referrals, emergency and slow triage, and linkage between upper and lower levels. The 2015 outline of the national health service system (2015-2020) puts forward the concept of “serious illness in hospital, minor illness in the community, rehabilitation back to the community”, emphasizing the need to expand the field of nursing to the family, community and society [10]. With the promotion of graded diagnosis and treatment system, under the background of high incidence of chronic diseases and heavy burden, more scholars have proposed to establish a hospital-community-family integrated management model. That is, a management system that brings chronic patients into the cooperation between the hospital and the community. Hospitals, communities and families are based on their own functions and positioning, with patients as the center. Information sharing and two-way referrals between tertiary hospitals and communities provide a comprehensive prevention and treatment model with full and continuous management services for patients in different courses of disease. At present, this model is mainly employed in the management of diabetes, stroke and other chronic diseases, and has achieved remarkable results [11]. Therefore, there is an urgent need to learn from some research experience, to explore a more scientific and effective management model of hypertension, to extend the management services of patients with hypertension from tertiary hospitals to communities and families, in order to achieve homogeneous management effect.

## 2. Patients and Methods

### 2.1. General Information

Sixty patients with hypertension treated in our hospital from July 2019 to July 2021 were enrolled.The patients were randomly divided into control group and study group. The former accepts routine management, while the latter accepts “hospital-community-family” integrated management. The age of the control group was 34-87 years, with an average of (65.78 ± 3.12) years, including 13 males and 17 females, while the study group was 34-88 years old, with an average age of (65.64 ± 3.55) years, including 15 males and 15 females. The general data have no statistical significance. With the permission of the Medical Ethics Association of our hospital, all patients signed the informed consent form.

Inclusion criteria: 1) all patients met the diagnostic criteria of the 2018 version of Chinese guidelines for Prevention and treatment of Hypertension [12]. The latest guidelines: systolic blood pressure (SBP) ≥140 mmHg and/or diastolic blood pressure (DBP) ≥90 mm Hg2) voluntarily participated in this study; 2) the age of the patients was more than 18 years old.

Exclusion criteria: 1) complicated with mental disorders or senile dementia; 2) complicated with liver and kidney diseases, malignant tumors or; 3) complicated with pregnancy or lactation; 4) complicated with congenital cardio-cerebrovascular diseases; 5) secondary hypertension; 6) patients with hypertension who refused to participate in this study after communication with members of the research team.

### 2.2. Treatment Methods

The control group carried out routine management: hypertension system health education, diet guidance, drug guidance, self-test, etc., and said that they had accepted relevant knowledge points at discharge and paid attention to patients' diet. In daily life, we should ensure adequate sleep time, dress loosely and comfortably, keep warm, and increase a certain amount of aerobic exercise.

The research group implemented the “hospital-community-family” trinity integrated management: 1) centralized visit: promote the relevant data, determine the patient's condition, confirm their lifestyle and eating habits, and establish personal health management files according to the patient's condition. Grasp the patient's condition, actively evaluate, explain the knowledge of hypertension-related diseases, and formulate a health management plan. The patients in the community were organized to teach centrally, imparted the knowledge related to hypertension, and made into a publicity manual, including the etiology and prognosis of hypertension, the role of antihypertensive drugs and matters needing attention, and the importance of taking medicine regularly. And instruct the patients how to use the sphygmomanometer, and tell them to measure the time and frequency correctly, and give demonstration education to the community staff, consult the relevant guidance measures to ensure that the patients can master the knowledge of hypertension. 2) telephone follow-up: a special telephone follow-up team was set up to regularly follow up the patients with hypertension in the community. The main purpose is to control the patients' blood pressure, their physical condition during the medication period, care about the patients' mental state, and guide the patients to develop good living habits. And praise the patients with good behavior in strict accordance with the doctor's advice, correct and understand the patients with poor medication, and help patients standardize the use of drugs; 3) door-to-door follow-up: door-to-door follow-up needs to accurately understand the situation of patients, check patients' physique and blood pressure, understand the changes of patients' blood pressure, encourage patients to ask questions, and build confidence for patients. Communicate with patients' families, assist patients with standardized medication, appropriate training, guide diet and rest, promote healthy diet, and ensure adequate sleep. At the same time, for patients with poor mood, timely psychological counseling, guide patients to actively face treatment, encourage patients to say the causes of bad mood, nurses actively carry out psychological counseling.

### 2.3. Observation Index

#### 2.3.1. Satisfaction

After consulting the literature and expert discussion, we designed patients' follow-up satisfaction, a total of 10 items, and recorded patients' satisfaction with follow-up management mode, health education, medical and nursing service, appointment registration process [13]. It is assigned into four dimensions: very satisfied, satisfied, general and dissatisfied. Satisfaction rate = very satisfaction rate + satisfaction rate + general rate.

#### 2.3.2. Blood Pressure Level

Blood pressure levels (diastolic blood pressure, systolic blood pressure) were measured with a sphygmomanometer before and 6 months after management.

#### 2.3.3. Disease Awareness Rate

A general questionnaire was adopted to investigate the awareness rate of hypertension related knowledge in the two groups 6 months after management, including hypertension related knowledge, hypertension harmfulness, community management methods, regular reexamination and blood pressure monitoring, etc., with a total score of 100, >90 as knowing, 70-90 as general awareness, <70 as not knowing [14].

#### 2.3.4. Anxiety and Depression Score

Evaluated by SDS and SAS scale [15]. The SDS scale included 20 items, each of which was evaluated by a 4-grade scale of 1-4 points, with 50 points as the boundary, <50 points for no depression, 50-60 points for mild depression, 60-70 points for moderate depression and>70 points for severe depression. The SAS scale also takes 50 points as the limit, less than 50 points as normal, 50-60 points as mild, 61-70 points as moderate, and>70 points as severe.

#### 2.3.5. Disease Control Ability

Based on the theory of self-management, combined with expert advice and actual situation, we developed a self-management questionnaire for patients with hypertension to understand the status of self-management in patients' daily diet and medication. Life. The questionnaire consists of 24 items, including diet management, medication management, behavior management and information management [16]. The questionnaire was evaluated by Likert 5 scale, with a score of 1-5 corresponding to “never, rarely, sometimes, often, always”, that is, “never =1, rarely =2, sometimes = 3, often = 4, always = 5”. Nine of the entries (T4 ~ T8, T11, T19 ~ T21) are reverse scores, that is, “never = 5 points, rarely = 4 points, sometimes = 3 points, often =2 points, always =1 points”. The lowest score of the questionnaire is 24, and the highest score is 120. The higher the score, the better the patient's self-management. The Cronbach *α* coefficient was 0.80, and each Cronbach *α* coefficient was more than 0.77. After two rounds of expert consultation, the content validity (I-CVI) of all items was more than 0.85. The overall content validity index (S-CVI) was 0.90. The reliability and validity of the questionnaire are good.

#### 2.3.6. Quality of Life Scale

The quality-of-life scale consists of four subscales, including physical, psychological, social and health self-awareness, with a total of 29 items [17]. The Cronbach's *α* coefficient of the scale is 0.79 to 0.91. The scale uses a 1-5 rating scale, and the lower the score, the higher the satisfaction.

### 2.4. Statistical Analysis

All the questionnaire data and score data were entered for the second time, and the data were statistically analyzed by SPSS 21.0 statistical software (Chinese version). All the data are in accordance with the normal distribution, and the measurement data are expressed by mean ± standard deviation (±s), using t-test; for repeated data measurement, the analysis of variance of repeated measurement data is adopted; the counting data rate n (%) is expressed by *χ* 2 test. P <0.05 indicates that the difference is statistically significant.

## 3. Results

### 3.1. Comparison of Nursing Satisfaction

First of all, we compared the nursing satisfaction: the study group was very satisfied in 25 cases, satisfactory in 4 cases, general in 1 case, and the satisfaction rate was 100.00%; in the control group, 10 cases were very satisfied, 8 cases were satisfied, 7 cases were general, and 5 cases were dissatisfied. The satisfaction rate was 83.33%. Compared to the control group, the nursing satisfaction of the study group was higher than that in control group (P <0.05). All the data results are indicated in figure 1.

### 3.2. Blood Pressure Level Comparison

Secondly, we compared blood pressure levels. There was no significant difference before management (P >0.05). Blood pressure decreased after treatment, and the level of blood pressure in the study group was lower than that in the control group (P <0.05). All the data results are indicated in figure 2.

### 3.3. Comparison of Disease Awareness Rate

Thirdly, we compared the rate of disease awareness. The scores of hypertension related knowledge, hypertension harmfulness, community management methods, regular reexamination and blood pressure monitoring in the study group were higher than those in the control group (P <0.05). All the data results are indicated in Table 1.

### 3.4. Comparison of Anxiety and Depression Scores

Next, compare anxiety and depression scores. There was no significant difference before management (P >0.05). The score of anxiety and depression in the study group was lower than that in the control group (P <0.05). All the data results are indicated in Table 2.

### 3.5. Comparison of Disease Control Ability

Then, we compared the ability of disease control. The total scores of diet management, drug management, behavior management and information management in the study group were higher than those in the control group (P <0.05). All the data results are indicated in Table 3.

### 3.6. Comparison of Quality of Life Scores

Finally, we compared the scores of quality of life. There was no significant difference before management (P >0.05). The scores of physiological function, psychological function, social function and health self-cognition in the study group were lower than those in the control group (P <0.05). All the data results are indicated in Table 4.

## 4. Discussion

Our results suggested that the nursing satisfaction of “hospital-community-family” integrated management was upregulated in comparison with routine management. Then, the level of blood pressure after “hospital-community-family” integrated management was considerably lower than that after routine management. After “hospital-community-family” integrated management, disease awareness rate of patients in study group was obviously enhanced than that after routine management. Patients experience more significant relief from anxiety and negative emotions following “hospital-community-family” integrated management so as to improved life quality.

Hypertension is a major public health problem worldwide [16]. According to the China Cardiovascular report, the prevalence rate of hypertension among adults in China is as high as 25.2%, and the estimated number of patients has reached 270 million [17]. Hypertension can cause severe target organ damage. Common complications include stroke, heart disease, kidney disease, peripheral vascular disease and fundus disease. About 70% of strokes and 50% of myocardial infarction are associated with high blood pressure. Once hypertension occurs with serious complications such as heart, brain and kidney, it becomes the leading cause of death from cardio-cerebrovascular diseases.At least half of the 3 million cardiovascular deaths each year are related to hypertension. Hypertension not only has a high rate of disability and mortality, but also seriously consumes medical and social resources, and its direct economic expenditure accounts for about 6.61% of the total health expenditure, bringing a heavy burden to families and countries [18]. The awareness rate, treatment rate and control rate of hypertension in people over 18 years old in China are 46.5%, 41.1% and 13.8%, respectively, which is still at a low level, and there is a large gap compared with developed countries [19]. Hypertension usually has no self-conscious symptoms, patients are easy to be ignored, can not be completely cured, and need lifelong management. Adhering to a healthy lifestyle and taking antihypertensive drugs are the main methods for the treatment of hypertension, both of which are indispensable. A healthy lifestyle is the foundation, and rational drug use is the key to achieving blood pressure standards. The two must be combined in order to effectively control hypertension. Studies have indicated that strengthening the supervision and management of patients with hypertension plays an important role in long-term control of blood pressure, reduction of clinical complications and target organ damage [20]. Therefore, strengthening the management of patients with hypertension is of great significance to promote the prognosis of patients.

For the management of hypertension, some countries mainly rely on the advantages of graded diagnosis and treatment, the United Kingdom, the United States and Canada and other countries have more mature management experience [21]. Graded diagnosis and treatment refers to the classification of diseases according to the degree of light, severe, slow, urgent and difficult. Medical institutions of different levels undertake the treatment of different levels of diseases, with a clear division of labor and reasonable medical treatment [21]. Primary health care services, namely grass-roots community health service institutions, secondary and tertiary medical services refer to specialist hospitals or general hospitals, as well as some teaching hospitals with first aid and major and difficult diseases as their main business [21, 22]. Each medical system is managed layer by layer, and the division of labor is clear. Meanwhile, a perfect regional medical information network system is established to connect personal health records, electronic medical records and hospitals, so as to realize the interconnection of networks among diagnosis and treatment institutions. Ensure smooth division of labor and cooperation and two-way referrals [22]. The community health service pays attention to all the residents of the community, carries on the disease health management to the hypertensive patients, 90% of the patients receive diagnosis and treatment in the primary health care system, and do not need to be referred to the superior organization, and the community general practitioner acts as the “gatekeeper”. Thus, It can be seen that the daily management of hypertension in western developed countries is mainly concentrated in the community, with the community as the main prevention and control to implement the management of chronic diseases such as hypertension [23].

The models of community management of hypertension in some countries mainly include chronic disease care model, chronic disease self-management model, continuous nursing model, peer support management model [24]. In the community, doctors, nurses, pharmacists and other team members use clinical information systems to provide evidence-based decision support for patients, and ultimately improve patients' self-management ability [24, 25]. In addition to doctors, the team also emphasizes that nurses and pharmacists are involved in the management of high blood pressure as health care managers. At present, the control rate of hypertension in the United States has reached 50% [25]. In addition to patients' health assessment, complications examination and health education, when patients are at high risk of disease, they need to be referred to appropriate medical services. The blood pressure level of more people receiving managed treatment is under control, and the blood pressure control rate in the UK has reached (63.0 ± 1.7) % as of 2011 [26]. Some experience indicates that the chronic disease care model is guided by the concept of graded diagnosis and treatment, based on nurses' health education, doctors deal with the abnormal value of blood pressure, and cooperate with multi-disciplinary teams. And with the help of the network platform to continuously evaluate patients' treatment compliance and drug plans, so that the treatment of a more individual telemedicine service is feasible and effective [27].

The traditional management methods implemented in our country include hierarchical management, self-management, family management and contract management. The trinity management of “hospital-community-family” is a new management mode, which means that the community health service center + secondary hospital + tertiary hospital forms a medical union, which can obtain preferential facilities from the aspects of medical treatment, referral, medication and medical insurance [28]. Different management methods have their own advantages and disadvantages, as follows: (1) hierarchical management: establishing health files of people's condition, grading and stratifying the disease severity of patients with hypertension, and taking corresponding measures according to different levels and layers, through regular follow-up and monitoring of patients. It can dynamically understand the changes of patients' blood pressure level, so as to realize two-way referral. Some scholars have indicated that grading management can take hypertension patients as objects, classify patients, make use of existing medical resources, and consciously grade intervention, so as to promote the blood pressure control rate and awareness rate; (2) self-management: self-management refers to hypertension patients with the assistance of community medical staff, through a series of health education courses to let patients know more knowledge, skills and confidence, can help patients build confidence in overcoming the disease, reduce the workload as much as possible, and give full play to the subjective initiative and matching degree of patients. Therefore, self-management can make up for the shortcomings and disadvantages of hierarchical management, and can rely on patients and their families to actively participate in it; (3) family management: family management is very important, this is a two-way management, family-based, supplemented by doctors. Doctors can make reasonable and comprehensive intervention programs according to the level and changes of patients' blood pressure, so that patients can understand the knowledge of hypertension, correctly guide their life and diet, and realize the prevention and treatment of hypertension. Clinical studies have shown that family management intervention can fully mobilize the strength of the family, help patients develop good living habits, and ultimately improve patients' treatment compliance and self-efficacy; (4) contract management: contract management is that hypertension patients and medical staff in the community further clarify the responsibilities and obligations of doctors and nurses through the community platform according to the voluntary principle and follow certain agreements, and formulate a targeted management plan according to the situation of patients. In order to achieve the desired management objectives. Previous studies have indicated that contract management can build a good doctor-patient relationship, help to improve patient management compliance, stabilize blood pressure, and change patients' bad living habits [29].

Changes in diet structure and lack of exercise brought about by some economic developments have led to a high incidence of hypertension, the most common chronic disease [29]. With the attention of the public to health, modern hypertension patients' excessive anxiety about their own health status, coupled with the serious complications of the disease, will affect the health and life of patients. At present, the management of hypertension in community is mainly based on the traditional management mode and the comprehensive management of the trinity of hospital, community and family [30]. The trinity integrated management of hospital-community-family is obviously more effective in the control of blood pressure and the reduction of complications. Clinically, every community doctor can actively carry out contract management on patients with hypertension and control them from the grass-roots level so as to achieve the goal of achieving blood pressure standards. The medical team, which is composed of family doctors, community nurses, public health doctors and volunteers, provides continuous health management services for patients through the mode of responsibility service. The “hospital-community-family” trinity integrated management model was first put forward in the guidance on promoting Family Doctor contract Service in June 2016, and with the deepening of the reform of the medical system, clinical management of chronic diseases has entered an era of prediction, prevention, individualized treatment and two-way referrals, which can not only meet the health needs of community residents in chronic disease management. The responsibility system of family doctors has become an important part of the comprehensive reform of community health and become the focus of the current research, and the application of family doctor responsibility system in patients with hypertension in the community is also the focus of attention [31]. In recent years, the family doctor responsibility system has been newly reported in the management of chronic diseases in the community, and achieved good results. The trinity comprehensive management of “hospital-community-family” is a new management model, which is the basis and the best choice for hypertension management. However, the management quality of patients with hypertension in the community is also affected by many factors, and the formulation of management methods should be considered and improved in many aspects and dimensions (1) Combined with the professional skills of community doctors, the professional skills training of community doctors should be strengthened, including their own professional skills, follow-up and communication skills, so as to continuously improve their own professional skills, improve patients' treatment compliance and build a good doctor-patient relationship; (2) continuously expand the number of doctors, while ensuring the number of community doctors, strengthen their management quality, let doctors and nurses master the latest management methods, and continuously improve the management quality; (3) be good at introducing new management models, actively carry out patients' self-activities, and carry out corresponding courses according to the characteristics of hypertension. With the help of Internet and multimedia technology, we should constantly update and develop new APP ports, strengthen patients' health education, change patients' bad habits and behaviors, and promote patients' awareness of self-prevention, so as to form a correct behavior and persevere, and enhance patients' survival and quality of life; (4) make full use of the medical resources of secondary and tertiary hospitals, set up chronic disease studios, and regularly consult grass-roots communities and community doctors under experts from secondary and tertiary hospitals, so as to provide high-quality and scientific management for patients. Existing practice data show that the implementation of “hospital-community-family” integrated management can significantly enhance the non-drug treatment of hypertension patients in the community. The hypertension management intervention effect of the family doctor contract model is better than the current community hypertension prevention and control follow-up management model. The same line of thinking can also be found in the study proposed by Noor A [32]. They applied new methods in their research, and their conclusions can also provide some support for this research.

Conclusively, adopting the comprehensive management of “hospital, community and family” trinity can vertically integrate medical resources and establish a truly effective hierarchical diagnosis and treatment model. At the same time, it takes advantage of the technical advantages of tertiary traditional Chinese medicine hospitals and highlights the management characteristics in the management content of the platform, which not only allows patients to Get full, seamless management to promote patient medication compliance and blood pressure control. It also enables community health care workers to improve their professional knowledge and skills. “Hospital-community-family” integrated management can promote patients' blood pressure and treatment compliance, enhance patients' self-management ability and self-confidence, and enhance the management efficiency of medical staff. Positive attitudes and high satisfaction among patients and medical staff.

## Figures and Tables

**Figure 1:** Comparison of nursing satisfaction between two groups.

**Figure 2:** Comparison of blood pressure level between two groups of patients.

**Table 1:** Comparison of disease awareness rate between the two groups[±s, Points].

Group	N	Knowledge related to hypertension	Hypertension harmfulness	Community management method	Regular review	Blood pressure monitoring
C group	30	81.29 ± 2.42	80.59 ± 2.34	79.59 ± 3.31	80.67 ± 2.31	83.95 ± 3.31
R group	30	94.19 ± 2.44	95.12 ± 1.21	93.67 ± 1.77	92.77 ± 1.67	95.12 ± 1.22
*t*		20.560	30.210	20.545	23.250	17.343
*P*		<0.01	<0.01	<0.01	<0.01	<0.01

**Table 2:** Comparison of anxiety and depression scores between the two groups [±s, Points].

Group	N	Anxiety score		Depression score	
		Before management	After management	Before management	After management
C group	30	69.94 ± 3.41	46.48 ± 1.44	70.79 ± 4.11	47.54 ± 3.34
R group	30	69.59 ± 3.45	41.29 ± 1.21	70.31 ± 4.56	38.79 ± 3.11
*t*		0.395	15.113	0.428	10.501
*P*		>0.05	<0.01	>0.05	<0.01

**Table 3:** Comparison of disease control ability between the two groups [±s, Points].

Group	N	Diet management	Medication management	Behavior management	Information management	Total score
C group	30	35.39 ± 2.45	11.69 ± 3.21	23.62 ± 2.45	5.79 ± 1.21	72.94 ± 1.35
R group	30	45.29 ± 1.21	18.59 ± 1.53	26.79 ± 1.26	10.38 ± 1.55	95.26 ± 3.11
*t*		19.844	10.627	6.302	12.785	36.058
*P*		<0.01	<0.01	<0.01	<0.01	<0.01

**Table 4:** Comparison of quality of life scores between the two groups before treatment [±s, Points].

Group	N	Physiological function		Psychological function		Social function		Healthy self-cognition	
		Before management	After management	Before management	After management	Before management	After management	Before management	After management
C Group	30	15.55 ± 4.63	13.13 ± 2.55	16.74 ± 3.52	14.42 ± 4.74	18.44 ± 3.31	16.42 ± 2.85	15.55 ± 3.16	13.86 ± 1.56
R group	30	15.64 ± 4.65	11.52 ± 2.53	16.52 ± 3.41	12.13 ± 1.58	18.56 ± 3.41	12.65 ± 3.12	15.56 ± 3.17	10.64 ± 2.55
*t*		0.075	2.454	0.245	2.510	0.138	4.886	0.012	5.889
*P*		>0.05	<0.01	>0.05	<0.01	>0.05	<0.01	>0.05	<0.01

## Data Availability

The datasets used and analyzed during the current study are available from the corresponding author upon reasonable request.
